The article "Exosomes From Cancer-Associated Mesenchymal Stem Cells Transmit TMBIM6 to Promote the Malignant Behavior of Hepatocellular Carcinoma via Activating PI3K/AKT Pathway" was retracted in 2023. Reasons: compromised peer review; unreliable results or conclusions.

# Exosomes From Cancer-Associated Mesenchymal Stem Cells Transmit TMBIM6 to Promote the Malignant Behavior of Hepatocellular Carcinoma *via* Activating PI3K/AKT Pathway

**DOI:** 10.3389/fonc.2022.868726

**Published:** 2022-06-02

**Authors:** Chuzhi Shang, Mi Ke, Lin Liu, Cong Wang, Yufang Liu, Xin Zheng

**Affiliations:** ^1^Department of Hepatobiliary Surgery, The First Affiliated Hospital of Xi’an Jiaotong University, Xi’an, China; ^2^Department of General Surgery, Shangzhou Regional Hospital, Shangluo, China

**Keywords:** hepatocellular carcinoma, cancer-associated mesenchymal stem cells, exosomes, TMBIM6, cancer progression

## Abstract

**Objective:**

Cancer-associated mesenchymal stem cells (MSCs) regulate the progression of cancers through exosome-delivered components, while few studies are conducted on hepatocellular carcinoma (HCC). This study aimed to evaluate the effect of exosomes from HCC-associated MSCs (HCC-MSCs) on HCC cellular functions and the potential regulatory mechanism.

**Methods:**

HCC cells (Huh7 and PLC) were cultured normally or co-cultured with HCC-MSCs, HCC-MSCs plus GW4869, or HCC-MSC-derived exosomes; then mRNA sequencing and RT-qPCR validation were conducted. Subsequently, candidate genes were sorted out and modified in HCC cells. Next, TMBIM6-modified HCC-MSCs were used to treat HCC cells.

**Results:**

Both HCC-MSCs and their derived exosomes promoted proliferation, invasion, sphere formation ability but suppressed apoptosis in HCC cells (all *p* < 0.05); however, the effect of HCC-MSCs on these cellular functions was repressed by exosome inhibitor (GW4869). Subsequently, TMBIM6, EEF2, and PRDX1 were sorted out by mRNA sequencing and RT-qPCR validation as candidate genes implicated in the regulation of HCC cellular functions by HCC-MSC-derived exosomes. Among them, TMBIM6 had a potent effect (all *p* < 0.05), while EEF2 and PRDX1 had less effect on regulating HCC cell viability and invasion. Next, direct silencing TMBIM6 repressed viability, sphere formation, invasion, epithelial–mesenchymal transition (EMT), and PI3K/AKT pathway but promoted apoptosis in HCC cells; however, overexpressing TMBIM6 showed the opposite effect. Furthermore, incubating with exosomes from TMBIM6-modified HCC-MSCs presented a similar effect as direct TMBIM6 modification in HCC cells.

**Conclusion:**

HCC-MSC-derived exosomes transmit TMBIM6 to promote malignant behavior *via* PI3K/AKT pathway in HCC.

## Introduction

Hepatocellular carcinoma (HCC) is one of the most fatal malignancies that cause more than 830,000 cases of deaths in 2020 worldwide according to a report from the WHO (1). Apart from that, with the increase in abuse of alcohol and the prevalence of non-alcoholic fatty liver disease, HCC is becoming a huge threat to the health of human beings (2–4). Considering the prevalence of hepatitis B virus infection in China, HCC is also one of the top dangers in China (5). Currently, the application of small molecular inhibitors, immune checkpoint inhibitors, and new technologies in locoregional therapy has improved the prognosis of HCC patients to some extent (6–9). However, there lacks a deep understanding of the detailed pathogenesis of HCC, which restricts the development of novel therapeutic agents for HCC.

Recently, the tumor microenvironment is regarded as a critical regulator of cancers, among which cancer-associated mesenchymal stem cells (CA-MSCs) have drawn wide attention considering their promotion of tumor progression in various cancers (10–12). For instance, MSCs derived from lung cancer facilitate invasion of lung cancer cells probably through inducing epithelial–mesenchymal transition (EMT) and increasing stemness-like properties in lung cancer cells (13). Meanwhile, gastric cancer-associated MSCs secrete hepatocyte growth factors to promote gastric cancer proliferation and metastasis *via* c-Myc-hexokinase 2 signaling (14). Besides, several studies confirm that ovarian cancer-associated MSCs enhance chemoresistance in ovarian cancer in multiple ways, including platelet-derived growth factor signaling, bone morphogenetic protein 4/hedgehog signaling loop, and phosphoinositide 3-kinase (PI3K)/protein kinase B (AKT) pathway (15–17). In HCC, several ways have been recognized to be implicated in HCC progressions promoted by HCC-associated MSCs (HCC-MSCs), such as long non-coding RNA (lncRNA) dynamin 3 opposite strand/lysine demethylase 6B/T-cell lymphoma invasion and metastasis-inducing protein 1 axis, lncRNA MSC-upregulated factor, and S100 calcium-binding protein A4/microRNA-155/suppressor of cytokine signaling 1/matrix metalloproteinase 9 axis (18–20). However, the regulation mechanism in HCC-MSCs facilitating HCC progression remains largely obscure.

The exosome is a vital intermediary that mediates cell–cell communication through transmitting its encapsulated contents, including RNA, DNA, protein, and lipid, thus participating in various biological processes, such as cancer progression (21–23). Regarding the regulation of exosomes in HCC progression, preceding studies have reported that exosomes secreted by high metastatic HCC cells, M2 macrophages, or MSCs exert either promotion or obstruction in HCC progression, mainly depending on the origin of exosomes (24–26). Exosomes and their contents are also regarded as predictive biomarkers for HCC prognosis (27, 28). Therefore, it is reasonable to deduce that HCC-MSC-derived exosomes may enhance HCC progression by transmitting the contents.

The current study aimed to investigate the implication of exosomes in HCC-MSC-mediated HCC malignant cellular functions, as well as the potential regulation approach.

## Methods

### Hepatocellular Carcinoma Tissues and Cell Culture

HCC tissues were obtained from patients at our hospital after approval by the Ethics Committee. Huh7 and PLC HCC cell lines were purchased from American Type Culture Collection (Manassas, VA, USA). All cells were cultured in α-MEM (Sigma, St. Louis, MO, USA) or Dulbecco’s modified Eagle’s medium (DMEM) (Sigma, USA) with 10% exosome-depleted fetal bovine serum (FBS) (Gibco, Grand Island, NY, USA) at 37°C with 5% CO_2_.

### Isolation and Characterization of Hepatocellular Carcinoma Mesenchymal Stem Cells

HCC-MSCs were extracted from HCC tissues as previously reported (20). Briefly, HCC tissues were minced and then dissociated with 0.1% collagenase (Gibco, USA) at 37°C for 1 h. The single-cell suspension was cultured with α-MEM containing 10% FBS and 1 ng/ml of bFGF (Gibco, USA) in non-coated polystyrene culture flasks (Corning, New York, NY, USA). HCC-MSCs were isolated based on the difference in the ability to adhere to plastic as fibroblast-like cells. Non-adherent cells were removed after 24 h, and the adherent fibroblast-like cells were cultured until 80% confluence. To identify the purity of MSCs, the cells were incubated with fluorescein isothiocyanate (FITC) Mouse Anti-Human CD34 (1:50, BD Biosciences, San Jose, CA, USA), CD44 (1:50, BD, USA), CD45 (1:50, BD, USA), CD73 (1:50, BD, USA), CD90 (1:50, BD, USA), and CD105 (1:50, BD, USA) antibodies. Then the cells were analyzed with a FACSCalibur flow cytometer (BD, USA).

### Isolation of Mesenchymal Stem Cell Exosomes

MSCs were cultured in the complete medium until they reached 80% confluence. Then, the culture medium was replaced by the serum-free medium. After 24-h culture, the exosomes from the culture medium of MSCs were extracted with a Total Exosome Isolation kit (Invitrogen, Carlsbad, CA, USA) according to the manufacturer’s instructions. The exosomes were quantified using Pierce bicinchoninic acid (BCA) Protein Assay Kit (Thermo Fisher Scientific, Waltham, MA, USA). Measurement of the exosome particle number was performed by Nanoparticle Tracking Analysis (NTA) using the NanoSight NS300 system (Malvern Instruments, Malvern, UK). Western blotting was performed to detect exosome marker proteins, including CD63, CD81, CD9, and Alix. The medium without culturing with MSCs was applied as negative control (NC).

### Co-Culture System

For inhibition of exosome generation, MSCs were treated with a culture medium containing 10 μM of GW4869 for 24 h (Sigma, USA) and marked as MSC-GW. Next, HCC cell co-culturing with MSCs, MSC-GW cells, or MSC exosomes was conducted with a transwell co-culture system (Corning, USA) based on a previous study (29). In brief, the HCC cells were seeded into the lower chamber. Then the MSCs or MSC-GW cells were seeded into the upper chamber and co-cultured with HCC cells. MSC exosomes were added into the upper chamber with the isovolumetric medium. The cultured Huh7 and PLC cells were divided into four groups: normal group (without any treatment), MSC group (co-cultured with MSCs), MSC-GW group (co-cultured with MSC-GW), and MSC-Exo group (co-cultured with 20 μg/ml of MSC exosomes). PKH-67 (Sigma, USA) staining was carried out to observe exosome uptake of Huh7 and PLC according to the manufacturer’s instructions. Huh7 and PLC cells were collected for proliferation, apoptosis, invasion, sphere formation, and RT-qPCR assays. Huh7 cells were harvested for RNA sequencing (RNA-seq).

### RNA Sequencing and Bioinformatics Analysis

The mRNA expression pattern of Huh7 cells from the above four groups and MSC exosomes were analyzed by RNA-seq. RNA-seq libraries were prepared using the TruSeq Stranded Total RNA Preparation kit (Illumina, San Diego, CA, USA) followed by sequencing on the Illumina HiSeq 2000 platform at Genergy Biotechnology (Shanghai, China). Data processing, principal component analysis (PCA), heatmap, differentially expressed gene (DEG), volcano plot, and Venn diagram were analyzed using R-project (Version 3.6.3). Gene Ontology (GO) and Kyoto Encyclopedia of Genes and Genomes (KEGG) pathway enrichment in DEGs were performed by DAVID (https://david.ncifcrf.gov/). The corresponding upregulated DEGs in the comparison of MSC_Exo vs. Normal and MSC vs. MSC_GW and high expression gene of MSC exosomes (Top 500) were analyzed by the Venn diagram and ranked by the average log_2_FC.

### Transfection Experiment in Hepatocellular Carcinoma Cells

A total of 50 nM of siRNA of transmembrane BAX inhibitor motif containing-6 (TMBIM6) (si-TMBIM6), EEF2 (si-EEF2), PRDX1 (si-PRDX1), and siRNA control (si-Ctrl) were obtained from Sangon (Shanghai, China) and transfected into Huh7 and PLC cells using HilyMax (Dojindo, Tokyo, Japan) according to the protocol. Cells were harvested for RT-qPCR, Western blotting, proliferation, and invasion assays after transfection.

### TMBIM6 Regulation Experiment of Hepatocellular Carcinoma Cells

The overexpression plasmids of TMBIM6 (oe-TMBIM6) and control plasmids (oe-Ctrl) were obtained from GenePharma Co., Ltd. (Shanghai, China). A total of 50 nM of si-TMBIM6 and si-Ctrl and 0.8 μg of oe-TMBIM6 and oe-Ctrl were transfected into Huh7 and PLC cells, respectively. After transfection, cells were harvested for RT-qPCR, Western blotting, proliferation, apoptosis, invasion, and sphere formation assays.

### Isolation of TMBIM6-Modified Mesenchymal Stem Cell Exosomes

After being transfected with si-TMBIM6, si-Ctrl, oe-TMBIM6, and oe-Ctrl, MSCs were cultured for 48 h, and then the culture medium was replaced by the serum-free medium. After 24-h culture, the exosomes from the culture medium of each group were extracted. RT-qPCR was performed for assessment of TMBIM6 expression in MSC and MSC exosomes after transfection.

### Hepatocellular Carcinoma Cell Culture With TMBIM6-Modified Mesenchymal Stem Cell Exosomes

Huh7 and PLC cells were cultured and divided into six groups: normal group (without any treatment), blank-Exo group (cultured with exosomes of normal MSCs), si-Ctrl-Exo group (cultured with exosomes of si-Ctrl MSCs), si-TMBIM6-Exo group (cultured with exosomes of si-TMBIM6 MSCs), oe-Ctrl-Exo group (cultured with exosomes of oe-Ctrl MSCs), and oe-TMBIM6-Exo group (cultured with exosomes of oe-TMBIM6 MSCs). After transfection, the RT-qPCR, Western blotting, proliferation, apoptosis, invasion, and sphere formation assays were carried out.

### Cell Proliferation, Apoptosis, Migration, and Invasion Assays

Cell Counting Kit-8 (Dojindo, Japan) was used for cell proliferation assay. Briefly, 2 × 10^3^ cells were seeded into 96-well plates. At 0, 24, 48, and 72 h after treatment, cells were incubated with 10 μl of reagent for 2 h. The optical density (OD) value was measured by SpectraMax^®^ 340 PC microplate reader (Molecular Devices, San Jose, CA, USA). Cell apoptosis assay was performed using a TUNEL apoptosis kit (Beyotime, Shanghai, China). Briefly, 4 × 10^4^ cells were seeded into 24-well plates. After 48-h treatment, cells were fixed, permeabilized, and then incubated with TUNEL reagent for 20 min, successively. Images were taken with a fluorescence microscope (Olympus, Tokyo, Japan). The apoptosis rate was calculated by the following formula: apoptosis cell (green) number/total cell (blue) number. Cell invasion assay was performed using Matrigel-coated transwell chambers (BD, USA). Briefly, after 48-h treatment, 5 × 10^4^ cells were plated into a transwell chamber and cultured for 24 h. After being fixed, the invasive cells were stained with crystal violet (Sangon, Shanghai, China). The number of invasive cells was counted under an inverted fluorescence microscope (Olympus, Japan). Cell migration was investigated by scratch wound assay. Briefly, a wound was scratched when the cells reach 80% confluence, followed by culturing for 24 h. Photos of the wound area were captured using an inverted microscope (Nikon, Melville, NY, Japan) at 0 and 24 h. The wound area was calculated using the Image‐Pro Plus 6.0 software (Media Cybernetics, Rockville, MD, USA).

### Sphere Formation Assay

For the co-culture system, MSCs or MSC-GW were seeded into the upper inserts. After culturing for 48 h, the inserts or MSC exosomes were added into the fresh wells of ultra-low attachment dishes (Corning, USA) filled with sphere medium and 1 × 10^3^ HCC cells. For TMBIM6-modified HCC cells, 1 × 10^3^ HCC cells were seeded into ultra-low attachment dishes after 48-h transfection. For HCC cells cultured with TMBIM6-modified MSC exosomes, 1 × 10^3^ HCC cells were seeded into ultra-low attachment dishes with a sphere medium containing exosomes from each group. Finally, all cells were incubated with DMEM/F12 medium (Gibco, USA) supplemented with 20 ng/ml of EGF (Gibco, USA), 10 ng/ml of bFGF, and 10 μl/ml of B27 (Gibco, USA) for 10 days. The number of spheres (diameter > 50 µm) was counted under a microscope (30).

### Reverse Transcriptase qPCR

Total RNA was prepared with TRIzol reagent (Invitrogen, Carlsbad, CA, USA). The cDNA was synthesized with PrimeScript™ RT reagent Kit (Takara, Maebashi, Japan). The PCR program was conducted with SYBR Premix Ex Taq™ (Takara, Japan). Results were calculated by the 2^−ΔΔCt^ method. The primers are listed in **Supplementary Table 1**.

### Western Blotting Assay

Total proteins were extracted with a lysis buffer (Sigma, USA) and quantified by a BCA Kit (Bio-Rad, Hercules, CA, USA). Proteins were separated using sodium dodecyl sulfate–polyacrylamide gel electrophoresis (SDS-PAGE) and transferred to nitrocellulose membrane (PALL, Port Washington, NY, USA). Next, the membranes were blocked with 5% bovine serum albumin (BSA) (Sigma, USA) for 1 h at 37°C and incubated overnight at 4°C with primary antibodies, followed by incubating with secondary antibodies (1:5,000, Abcam, Cambridge, UK) successively. The bands were visualized using an enhanced chemiluminescence (ECL) kit (Beyotime, China) and exposed to X-ray film (Carestream, Concord, ON, Canada). The antibodies are listed in **Supplementary Table 2**.

### Statistical Analysis

Statistical analyses were performed using GraphPad Prism 7.0 software. One-way ANOVA followed by Tukey’s or Dunnett’s multiple comparisons test was used for comparison between groups. *p* < 0.05 was considered statistically significant. * indicated *p* < 0.05; ** indicated *p* < 0.01; *** indicated *p* < 0.001; NS indicated not significant.

## Results

### Hepatocellular Carcinoma Mesenchymal Stem Cells and Their Derived Exosomes Promoted Hepatocellular Carcinoma Proliferation, Invasion, and Sphere Formation Ability

First of all, HCC-MSCs were isolated from primary HCC tissues. After culturing, the cells presented fusiform shape, highly expressing CD44, CD73, CD90, and CD105 while negatively expressing CD34 and CD45 (**Supplementary Figures 1A, B**), indicating the high purity of HCC-MSCs. Meanwhile, the exosomes of HCC-MSCs were isolated and identified (**Supplementary Figures 1C, D**). Moreover, HCC cells absorbed these exosomes when co-culturing with HCC-MSCs (**Supplementary Figure 1E**).

Subsequently, the effect of HCC-MSCs or their derived exosomes on HCC malignant cellular functions was investigated, which revealed that both co-culture of HCC-MSCs and their derived exosomes improved proliferation (**Figure 1A**), invasion (**Figures 1B, C**), and sphere formation ability (**Figures 1D, E**) while inhibiting apoptosis (**Figures 1F, G**) in Huh7 and PLC cells (all *p* < 0.05). However, when the generation of exosomes was suppressed *via* GW4869 treatment in HCC-MSCs, they had less effect on the abovementioned HCC malignant cellular functions (all *p* > 0.05) (**Figures 1A–G**). Besides, HCC-MSCs also promoted the migration of Huh7 and PLC cells (both *p* < 0.05) (**Supplementary Figures 2A, B**).

**Figure 1:** Effect of HCC-MSCs and their derived exosomes on HCC cellular functions. Comparison of viability **(A)**, invasion **(B, C)**, sphere formation ability **(D, E)**, and apoptosis **(F, G)** among groups in Huh7 and PLC cells. HCC cells were cultured normally or co-incubated by HCC-MSCs, HCC-MSCs with GW4869 treatment, or exosomes of HCC-MSCs. Purple cells indicate invaded cells in panel **(B)** Green cells indicate apoptotic cells in panel **(D)** NS, not significant; *p < 0.05; **p < 0.01. HCC, hepatocellular carcinoma; MSCs, mesenchymal stem cells.

### TMBIM6 Was a Potentially Key Gene Involved in Hepatocellular Carcinoma Mesenchymal Stem Cell Exosome-Mediated Regulation on Hepatocellular Carcinoma Cellular Functions

Next, RNA-seq and bioinformatics analysis were conducted in MSC-Exo vs. Normal groups and MSC vs. MSC-GW groups in HCC cells (**Supplementary Figures 3A-J**). A total of 217 upregulated and 162 downregulated DEGs were identified synchronously in MSC-Exo vs. Normal groups and MSC vs. MSC-GW groups (**Figure 2A**); GO and KEGG enrichment analyses revealed that these DEGs were mainly enriched in the molecular function of protein binding, cellular component of cytosol, the biological process of positive regulation of cell proliferation, and signaling pathways including PI3K/AKT, Wnt, and TGF-β pathways (**Supplementary Figure 4**). Moreover, 45 candidate DEGs, with TMBIM6, EEF2, and PRDX1 as the top 3, were sorted out among the intersection of upregulated DEGs in MSC-Exo vs. Normal groups, upregulated DEGs in MSC vs. MSC-GW groups, and top 500 highly expressed genes in HCC-MSC exosomes (**Figures 2B, C**). Then, RT-qPCR verified that TMBIM6, EEF2, and PRDX1 were upregulated in HCC cells when co-culturing with HCC-MSCs or their derived exosomes (all *p* < 0.05) (**Figure 2D**).

**Figure 2:** RNA sequencing and RT-qPCR validation. Venn diagram showing upregulated and downregulated DEGs between MSC_Exo versus normal groups and MSC versus MSC_GW group **(A)**. Venn diagram showing intersection among upregulated DEGs in MSC_Exo versus normal groups, upregulated DEGs in MSC versus MSC_GW group, and top 500 upregulated genes in exosomes of HCC-MSCs **(B)**. Total 45 genes in the intersection **(C)**. RT-qPCR validation of TMBIM6, EEF2, and PRDX1 among groups **(D)**. NS, not significant; *p < 0.05; **p < 0.01; ***p < 0.001. DEGs, differentially expressed genes; MSC, mesenchymal stem cell; HCC, hepatocellular carcinoma.

Further, TMBIM6, EEF2, and PRDX1 were knocked down by transfection of their respective siRNAs in HCC cells, whose transfection efficiencies were demonstrated by RT-qPCR and Western blotting (**Figures 3A–C**). Cell Counting Kit-8 (CCK-8 assay) and transwell assay revealed that TMBIM6 knockdown suppressed proliferation and invasion in Huh7 and PLC cells strongly (all *p* < 0.05), PRDX1 knockdown showed less effect, and EEF2 knockdown could not affect HCC cell proliferation or invasion (**Figures 3D–F**). Therefore, TMBIM6 was considered a potentially key modulator involved in the HCC-MSC exosome-mediated regulation of HCC cellular functions.

**Figure 3:** Effect of TMBIM6, EEF2, and PRDX1 on viability and invasion of HCC cells. Expressions of TMBIM6 **(A)**, EEF2 **(B)**, and PRDX1 **(C)** in Huh7 and PLC cells after transfection. Comparison of viability **(D)** and invasion **(E, F)** among groups in Huh7 and PLC cells. HCC cells were cultured normally or transfected with control, TMBIM6, EEF2, or PRDX1 siRNAs. Purple cells indicate invaded cells in panel **(E)** NS, not significant; *p < 0.05; **p < 0.01; ***p < 0.001. HCC, hepatocellular carcinoma.

### TMBIM6 Promoted Cell Proliferation, Invasion, Sphere Formation, Epithelial–Mesenchymal Transition, and PI3K/AKT Pathway in Hepatocellular Carcinoma

TMBIM6 was overexpressed or knocked down in Huh7 and PLC cells to explore its effect on HCC cellular functions through transfection of overexpression plasmid or siRNA, whose efficiencies were evaluated by RT-qPCR and Western blotting (**Figure 4A**). The subsequent experiments revealed that TMBIM6 knockdown suppressed proliferation (both *p* < 0.05), promoted apoptosis (both *p* < 0.05), inhibited sphere formation ability (only *p* < 0.05 in Huh7 cells but *p* > 0.05 in PLC cells), and reduced invasion (both *p* < 0.05) in Huh7 and PLC cells, while TMBIM6 overexpression exerted the opposite effect (all *p* < 0.05) (**Figures 4B–H**).

**Figure 4:** Effect of TMBIM6 on viability, apoptosis, sphere formation ability, and invasion of HCC cells. Expression of TMBIM6 in Huh7 and PLC cells after transfection **(A)**. Comparison of viability **(B)**, apoptosis **(C, D)**, sphere formation ability **(E, F)**, and invasion **(G, H)** among groups in Huh7 and PLC cells. HCC cells were cultured normally or transfected with control siRNA, TMBIM6 siRNA, control overexpression plasmids, or TMBIM6 overexpression plasmids. Green cells indicate apoptotic cells in panel **(C)** Purple cells indicate invaded cells in panel **(G)**. NS, not significant; *p < 0.05; **p < 0.01; ***p < 0.001. HCC, hepatocellular carcinoma.

Furthermore, TMBIM6 knockdown upregulated E-cadherin (both *p* < 0.05) but downregulated N-cadherin (both *p* < 0.05), vimentin (only *p* < 0.05 in PLC cells), and Slug (both *p* < 0.05) in Huh7 and PLC cells; however, TMBIM6 overexpression presented the inverse trends (all *p* < 0.05 except for E-cadherin in PLC cells) (**Figures 5A, B**). Since the PI3K/AKT pathway is a critical pathway that regulates multiple cellular functions and the progression of HCC, it was further investigated in this study. The phosphorylation of PI3K (only *p* < 0.05 in Huh7 cells) and AKT (both *p* < 0.05) was decreased by TMBIM6 knockdown but increased by TMBIM6 overexpression (all *p* < 0.05) in Huh7 and PLC cells (**Figures 5C, D**). These data indicated that TMBIM6 knockdown suppressed EMT and PI3K/AKT pathway in HCC cells, while TMBIM6 overexpression presented the opposite effect.

**Figure 5:** Effect of TMBIM6 on EMT markers and PI3K/AKT pathway in HCC cells. Comparison of EMT markers **(A, B)** and phosphorylation of PI3K and AKT **(C, D)** among groups in Huh7 and PLC cells. HCC cells were cultured normally or transfected with control siRNA, TMBIM6 siRNA, control overexpression plasmids, or TMBIM6 overexpression plasmids. NS, not significant; *p < 0.05; **p < 0.01. EMT, epithelial–mesenchymal transition; HCC, hepatocellular carcinoma.

### Exosomes From TMBIM6-Modified Hepatocellular Carcinoma Mesenchymal Stem Cells Regulated Cell Proliferation, Invasion, Sphere Formation, EMT, and PI3K/AKT Pathway in Hepatocellular Carcinoma

In order to further validate whether HCC-MSCs could regulate HCC malignant behaviors through transmitting TMBIM6 *via* exosomes, TMBIM6 was modified in HCC-MSCs. The transfection efficacy of TMBIM6 siRNA or overexpression plasmids in HCC-MSCs and their exosomes was reflected by RT-qPCR data (**Figures 6A, B**). Then the exosomes were isolated and cultured with HCC cells, which presented that TMBIM6 was accordingly regulated in Huh7 and PLC cells co-cultured with exosomes from TMBIM6-modified HCC-MSCs (all *p* < 0.05) (**Figure 6C**).

**Figure 6:** Effect of exosomes from TMBIM6-modified HCC-MSCs on viability, apoptosis, and sphere formation ability of HCC cells. Expression of TMBIM6 in HCC-MSCs **(A)** and their derived exosomes **(B)** after transfection. Expression of TMBIM6 in HCC cells after being co-cultured with exosomes from TMBIM6-modified HCC-MSCs **(C)**. Comparison of viability **(D)**, apoptosis **(E**, **F)**, and sphere formation ability **(G, H)** among groups in Huh7 and PLC cells. HCC-MSCs were cultured normally or transfected with control siRNA, TMBIM6 siRNA, control overexpression plasmids, or TMBIM6 overexpression plasmids; then HCC cells were cultured normally or co-cultured with exosomes from TMBIM6-modified HCC-MSCs. Green cells indicted apoptotic cells in **(E)** NS, not significant; *p < 0.05; **p < 0.01; ***p < 0.001. HCC, hepatocellular carcinoma; MSCs, mesenchymal stem cells.

Further experiments revealed that culturing with TMBIM6 knockdown exosomes reduced proliferation (both *p* < 0.05); increased apoptosis (both *p* < 0.05); suppressed sphere formation (both *p* < 0.05); inhibited invasion (both *p* < 0.05); promoted E-cadherin (both *p* < 0.05); repressed N-cadherin (both *p* < 0.05), vimentin (only *p* < 0.05 in Huh7 cells), and Slug (only *p* < 0.05 in PLC cells); and decreased phosphorylation of PI3K (both *p* < 0.05) and AKT (only *p* < 0.05 in PLC cells) in Huh7 and PLC cells (**Figures 6D–H**, **7A–F**). However, culturing with TMBIM6 overexpressed exosomes presented the reverse effect (all *p* < 0.05) as that of TMBIM6 knockdown exosomes did, although statistical significance was not observed in cell viability, apoptosis, and sphere formation ability in PLC cells (**Figures 6D–H**, **7A–F**).

**Figure 7:** Effect of exosomes from TMBIM6-modified HCC-MSCs on invasion, EMT markers, and PI3K/AKT pathway in HCC cells. Comparison of invasion **(A, B)**, EMT markers **(C, D)**, and phosphorylation of PI3K and AKT **(E, F)** among groups in Huh7 and PLC cells. HCC-MSCs were cultured normally or transfected with control siRNA, TMBIM6 siRNA, control overexpression plasmids, or TMBIM6 overexpression plasmids; then HCC cells were cultured normally or co-cultured with exosomes from TMBIM6-modified HCC-MSCs. Purple cells indicate invaded cells in panel **(A)**. NS, not significant; *p < 0.05; **p < 0.01. HCC, hepatocellular carcinoma; MSCs, mesenchymal stem cells; EMT, epithelial–mesenchymal transition.

## Discussion

The tumor microenvironment is a complex system composed of various cells, among which tumor cells recruit and educate the stromal cells (including immune cells, CA-MSCs, cancer-associated fibroblasts, etc.), and the latter ones regulate antitumor immune response and modulate tumor growth, metastasis, and drug resistance (9, 10). One of the key components that mediate intracellular communication in the tumor microenvironment is exosomes (31). For instance, it is reported that exosomes derived from melanoma cells increase the differentiation of human umbilical vein endothelial cells into cancer-associated fibroblasts, and the latter ones promote cancer progression (32). Another study discloses that exosomes derived from adenocarcinoma gastric cancer cells promote the migration and invasion of adipose-derived MSCs through transmitting circular RNA 0004303 (33). Regarding communication of CA-MSCs to other components of the tumor microenvironment *via* exosomes, it is reported that breast CA-MSCs induce differentiation of monocytic myeloid-derived suppressor cells into M2-polarized macrophages, which support breast cancer progression (34). Meanwhile, CA-MSCs also directly communicate to various cancer cells *via* exosomes. For example, CA-MSCs increase breast cancer cell proliferation and resistance to chemotherapeutic agents (35); CA-MSCs promote the migration of atypical teratoid/rhabdoid tumor cells through transferring exosomal miR-155 (36).

As mentioned earlier, although several previous studies have illustrated the regulation of HCC-MSCs on the progression of HCC (18–20), whether this regulation is dependent on the communication by exosomes remains unclear. In the current study, the data presented that the co-incubation of HCC-MSCs with HCC cell lines promoted proliferation, migration, sphere formation ability, and EMT but suppressed apoptosis of HCC cell lines, indicating that HCC-MSCs enhanced the progression of HCC, which was partly in line with previous reports (18–20). Furthermore, by using exosome inhibitor GW4869, it was disclosed that exosomes were necessary for the regulation of HCC progression by HCC-MSCs, which, to the best of our knowledge, had not been reported by other studies. However, several published studies display that exosomes from bone marrow MSCs impede the progression of HCC (25, 37, 38). The differences between the current study and those previous ones are because MSCs from different sources have different roles in cancer progression, in which CA-MSCs promote cancer progression while bone marrow MSCs exert the reverse effect.

In the current study, RNA-seq, bioinformatics analysis, and RT-qPCR validation were conducted, which might provide a comprehensive view of the potential molecular mechanism engaged in the regulation of HCC cell malignant functions by HCC-MSC-derived exosomes (39). The data revealed that 217 upregulated and 162 downregulated DEGs were closely related to the regulation of HCC cellular functions by HCC-MSC-derived exosomes. Meanwhile, KEGG enrichment revealed that these DEGs were mainly enriched in pathways including PI3K/AKT, Wnt, and TGF-beta pathways, which are well-recognized pathways that facilitate the malignant behavior of cancer cells, including HCC (40–42). Furthermore, TMBIM6, EEF2, and PRDX1 were filtered out from these DEGs. Although TMBIM knockdown suppressed proliferation and invasion of HCC cells, knockdown of EEF2 or PRDX1 had little or no effect on proliferation or invasion of HCC cells. However, previous studies have implied that EEF2 and PRDX1 participate in the progression of HCC (43, 44). The difference between the findings of this study and previous studies might be explained by different HCC cell lines. Therefore, we focused on TMBIM6 in the subsequent experiments.

TMBIM6, also known as Bax inhibitor-1, is an inhibitor of Bax-mediated apoptosis (45). In cancers, TMBIM6 is regarded as a promoter of cancer progression. For example, TMBIM6 regulates the extracellular signal-regulated kinase (ERK) pathway to promote the proliferation and migration of breast cancer cells (46). Another study reveals that TMBIM6 enhances proliferation and metastasis in non-small cell lung cancer cells (47). Other studies also report similar conclusions that TMBIM6 participates in the progression of laryngeal squamous cell carcinoma, glioblastoma, etc. (48, 49). However, whether TMBIM6 also facilitates the progression of HCC remains to be explored; besides, its involvement in the tumor microenvironment is not clear. In the present study, it was disclosed that TMBIM6 was transferred to HCC cells from HCC-MSCs *via* exosomes; meanwhile, this procedure promoted proliferation, migration, sphere formation ability, and EMT but suppressed apoptosis of HCC cells. Among the cellular functions, sphere formation ability and EMT are closely related to stemness, which is partly responsible for tumor progression, chemoresistance, and cancer relapse (50). However, no previous study has reported the regulation of TMBIM6 on cancer stemness. Our study implied that TMBIM6 might regulate stemness in HCC, while further studies should be conducted to verify this. The findings of our study highlighted the potential of HCC-MSC-derived exosomal TMBIM6 as a therapeutic target of HCC.

PI3K/AKT pathway is a classic signaling pathway that regulates multiple cellular functions including proliferation, migration, invasion, and stemness in cancers (51). Recent studies disclose that in HCC, PI3K/AKT pathway is activated by the exosomes from high metastatic HCC cells or macrophages *via* transmitting miRNAs (26, 52). In the present study, it was revealed that PI3K/AKT pathway in HCC cells could also be activated by HCC-MSC-derived exosomal TMBIM6. Therefore, it could be deduced that in HCC, PI3K/AKT pathway might be activated by various components of the tumor microenvironment. Studies in the future were encouraged to further explore this issue.

In the present study, HCC-MSCs were directly separated from HCC tissues. Although using HCC-MSCs from HCC tissues might better mimic the HCC microenvironment, which was one of the highlights of this study, some issues might be caused by this. For instance, it was possible that some matrix cells of HCC tissues were brought into the co-culture system between HCC cells and HCC-MSCs, which might slightly influence the results. Besides, our findings might be affected by the genetic characteristics of the HCC patients who donated HCC tissues for HCC-MSC isolation. Apart from that, our study only used two HCC cell lines; thus, the findings of this study should be verified in other HCC cell lines. Animal studies using the siRNA and overexpression plasmids of TMBIM6 should be conducted in the future. Further clinical validation should be conducted.

To conclude, HCC-MSC-derived exosomal TMBIM6 promotes proliferation, invasion, sphere formation ability, and EMT *via* activating PI3K/AKT pathway in HCC, indicating that it could be a potential treatment target for HCC.

## Data Availability Statement

The original contributions presented in the study are included in the article/**Supplementary Material**. Further inquiries can be directed to the corresponding author.

## Author Contributions

XZ conceived and designed the study. CS, MK, and LL performed the experiments. CW and YL analyzed and interpreted the data and drafted the manuscript. All authors participated in the writing and revision of the manuscript. All authors read and approved the final manuscript.

## Funding

This study was supported by grants from the National Natural Scientific Foundation of China (81301743 and 81572733 to XZ), Research Fund for the Doctoral Program of High Education of China from the Ministry of Education (No. 20120201120090 to XZ), New Medicine Research Project from THE First Hospital of Xi’an Jiaotong University (XJTU1AF-CRF-2016-002), Key Science and Technology Program of Shaanxi Province (Nos. 2014K11-01-01-21 and 2016SF-206 to XZ), and the Fundamental Research Funds for the Basic Research Operating Expenses Program of Central College sponsored by Xi’an Jiaotong University to XZ.

## Conflict of Interest

The authors declare that the research was conducted in the absence of any commercial or financial relationships that could be construed as a potential conflict of interest.

## Publisher’s Note

All claims expressed in this article are solely those of the authors and do not necessarily represent those of their affiliated organizations, or those of the publisher, the editors and the reviewers. Any product that may be evaluated in this article, or claim that may be made by its manufacturer, is not guaranteed or endorsed by the publisher.

## Supplementary Material

Supplementary Figure 1 Characterization of HCC-MSCs and their derived exosomes. HCC-MSCs under bright field **(A)**; surface markers of HCC-MSCs **(B)**; particle size analysis of HCC-MSCs derived exosomes **(C)**; exosome marker analysis **(D)**; observation of exosomes absorbed by HCC cells **(E)**.

Supplementary Figure 2 Effect of HCC-MSCs on migration of HCC cells. Representative images of migration detection **(A)**; Comparison of migration rate between groups **(B)**.

Supplementary Figure 3 RNA sequencing in Huh7 cells. PCA **(A)**, heatmap **(B)** and volcano plot (**C**) analyses between MSC_Exo group and normal group; GO **(D)** and KEGG **(E)** enrichment of DEGs between MSC_Exo group and normal group. PCA **(F)**, heatmap (**G**) and volcano plot **(H)** analyses between MSC group and MSC_GW group; GO **(I)** and KEGG **(J)** enrichment of DEGs between MSC group and MSC_GW group.

Supplementary Figure 4 GO and KEGG enrichment of DEGs between MSC_Exo versus normal groups and MSC versus MSC_GW group.

## References

[1] SungHFerlayJSiegelRLLaversanneMSoerjomataramIJemalA. Global Cancer Statistics 2020: GLOBOCAN Estimates of Incidence and Mortality Worldwide for 36 Cancers in 185 Countries. CA Cancer J Clin (2021) 71(3):209–49. doi: 10.3322/caac.21660 33538338

[2] IoannouGN. Epidemiology and Risk-Stratification of NAFLD-Associated HCC. J Hepatol (2021) 75(6):1476–84. doi: 10.1016/j.jhep.2021.08.012 34453963

[3] LoftfieldEStepienMViallonVTrijsburgLRothwellJARobinotN. Novel Biomarkers of Habitual Alcohol Intake and Associations With Risk of Pancreatic and Liver Cancers and Liver Disease Mortality. J Natl Cancer Inst (2021) 113(11):1542–50. doi: 10.1093/jnci/djab078 PMC856296934010397

[4] HuangDQEl-SeragHBLoombaR. Global Epidemiology of NAFLD-Related HCC: Trends, Predictions, Risk Factors and Prevention. Nat Rev Gastroenterol Hepatol (2021) 18(4):223–38. doi: 10.1038/s41575-020-00381-6 PMC801673833349658

[5] WangXKangMLiuCLinTHanXJiangX. Current State and Progress of Research on the Role of lncRNA in HBV-Related Liver Cancer. Front Cell Infect Microbiol (2021) 11:714895. doi: 10.3389/fcimb.2021.714895 34869051PMC8636595

[6] SchnitzbauerAAFilmannNAdamRBachellierPBechsteinWOBeckerT. mTOR Inhibition Is Most Beneficial After Liver Transplantation for Hepatocellular Carcinoma in Patients With Active Tumors. Ann Surg (2020) 272(5):855–62. doi: 10.1097/SLA.0000000000004280 32889867

[7] XuJZhangYJiaRYueCChangLLiuR. Anti-PD-1 Antibody SHR-1210 Combined With Apatinib for Advanced Hepatocellular Carcinoma, Gastric, or Esophagogastric Junction Cancer: An Open-Label, Dose Escalation and Expansion Study. Clin Cancer Res (2019) 25(2):515–23. doi: 10.1158/1078-0432.CCR-18-2484 30348638

[8] PinyolRMontalRBassaganyasLSiaDTakayamaTChauGY. Molecular Predictors of Prevention of Recurrence in HCC With Sorafenib as Adjuvant Treatment and Prognostic Factors in the Phase 3 STORM Trial. Gut (2019) 68(6):1065–75. doi: 10.1136/gutjnl-2018-316408 PMC658074530108162

[9] FacciorussoA. Drug-Eluting Beads Transarterial Chemoembolization for Hepatocellular Carcinoma: Current State of the Art. World J Gastroenterol (2018) 24(2):161–9. doi: 10.3748/wjg.v24.i2.161 PMC576893529375202

[10] XiaoYYuD. Tumor Microenvironment as a Therapeutic Target in Cancer. Pharmacol Ther (2021) 221:107753. doi: 10.1016/j.pharmthera.2020.107753 33259885PMC8084948

[11] MaoXXuJWangWLiangCHuaJLiuJ. Crosstalk Between Cancer-Associated Fibroblasts and Immune Cells in the Tumor Microenvironment: New Findings and Future Perspectives. Mol Cancer (2021) 20(1):131. doi: 10.1186/s12943-021-01428-1 34635121PMC8504100

[12] ZhangJJiCLiWMaoZShiYShiH. Tumor-Educated Neutrophils Activate Mesenchymal Stem Cells to Promote Gastric Cancer Growth and Metastasis. Front Cell Dev Biol (2020) 8:788. doi: 10.3389/fcell.2020.00788 32903528PMC7438587

[13] YanCChangJSongXQiYJiZLiuT. Lung Cancer-Associated Mesenchymal Stem Cells Promote Tumor Metastasis and Tumorigenesis by Induction of Epithelial-Mesenchymal Transition and Stem-Like Reprogram. Aging (Albany NY) (2021) 13(7):9780–800. doi: 10.18632/aging.202732 PMC806421933744858

[14] ChenBCaiTHuangCZangXSunLGuoS. G6PD-NF-kappaB-HGF Signal in Gastric Cancer-Associated Mesenchymal Stem Cells Promotes the Proliferation and Metastasis of Gastric Cancer Cells by Upregulating the Expression of HK2. Front Oncol (2021) 11:648706. doi: 10.3389/fonc.2021.648706 33718248PMC7952978

[15] CastellsMMilhasDGandyCThibaultBRafiiADelordJP. Microenvironment Mesenchymal Cells Protect Ovarian Cancer Cell Lines From Apoptosis by Inhibiting XIAP Inactivation. Cell Death Dis (2013) 4:e887. doi: 10.1038/cddis.2013.384 24176845PMC3824693

[16] CoffmanLGChoiYJMcLeanKAllenBLdi MaglianoMPBuckanovichRJ. Human Carcinoma-Associated Mesenchymal Stem Cells Promote Ovarian Cancer Chemotherapy Resistance *via* a BMP4/HH Signaling Loop. Oncotarget (2016) 7(6):6916–32. doi: 10.18632/oncotarget.6870 PMC487275826755648

[17] RaghavanSSnyderCSWangAMcLeanKZamarinDBuckanovichRJ. Carcinoma-Associated Mesenchymal Stem Cells Promote Chemoresistance in Ovarian Cancer Stem Cells *via* PDGF Signaling. Cancers (Basel) (2020) 12:(8). doi: 10.3390/cancers12082063 32726910PMC7464970

[18] WangWWangQHuangDBSunQKWuSSZhaoYJ. Tumor-Associated Mesenchymal Stem Cells Promote Hepatocellular Carcinoma Metastasis *via* a DNM3OS/KDM6B/TIAM1 Axis. Cancer Lett (2021) 503:19–31. doi: 10.1016/j.canlet.2021.01.011 33472090

[19] YanXZhangDWuWWuSQianJHaoY. Mesenchymal Stem Cells Promote Hepatocarcinogenesis *via* lncRNA-MUF Interaction With ANXA2 and miR-34a. Cancer Res (2017) 77(23):6704–16. doi: 10.1158/0008-5472.CAN-17-1915 28947421

[20] YanXLJiaYLChenLZengQZhouJNFuCJ. Hepatocellular Carcinoma-Associated Mesenchymal Stem Cells Promote Hepatocarcinoma Progression: Role of the S100A4-Mir155-SOCS1-MMP9 Axis. Hepatology (2013) 57(6):2274–86. doi: 10.1002/hep.26257 23316018

[21] IsaacRReisFCGYingWOlefskyJM. Exosomes as Mediators of Intercellular Crosstalk in Metabolism. Cell Metab (2021) 33(9):1744–62. doi: 10.1016/j.cmet.2021.08.006 PMC842880434496230

[22] TangXHGuoTGaoXYWuXLXingXFJiJF. Exosome-Derived Noncoding RNAs in Gastric Cancer: Functions and Clinical Applications. Mol Cancer (2021) 20(1):99. doi: 10.1186/s12943-021-01396-6 34330299PMC8323226

[23] NooninCThongboonkerdV. Exosome-Inflammasome Crosstalk and Their Roles in Inflammatory Responses. Theranostics (2021) 11(9):4436–51. doi: 10.7150/thno.54004 PMC797744833754070

[24] LiWXinXLiXGengJSunY. Exosomes Secreted by M2 Macrophages Promote Cancer Stemness of Hepatocellular Carcinoma *via* the miR-27a-3p/TXNIP Pathways. Int Immunopharmacol (2021) 101(Pt A):107585. doi: 10.1016/j.intimp.2021.107585 34601333

[25] MaYSLiuJBLinLZhangHWuJJShiY. Exosomal microRNA-15a From Mesenchymal Stem Cells Impedes Hepatocellular Carcinoma Progression *via* Downregulation of SALL4. Cell Death Discovery (2021) 7(1):224. doi: 10.1038/s41420-021-00611-z 34455417PMC8403170

[26] YangBFengXLiuHTongRWuJLiC. High-Metastatic Cancer Cells Derived Exosomal Mir92a-3p Promotes Epithelial-Mesenchymal Transition and Metastasis of Low-Metastatic Cancer Cells by Regulating PTEN/Akt Pathway in Hepatocellular Carcinoma. Oncogene (2020) 39(42):6529–43. doi: 10.1038/s41388-020-01450-5 PMC756149732917956

[27] ZhuJTangBGaoYXuSTuJWangY. Predictive Models for HCC Prognosis, Recurrence Risk, and Immune Infiltration Based on Two Exosomal Genes: MYL6B and THOC2. J Inflammation Res (2021) 14:4089–109. doi: 10.2147/JIR.S315957 PMC840302934466015

[28] DengPLiMWuY. The Predictive Efficacy of Serum Exosomal microRNA-122 and microRNA-148a for Hepatocellular Carcinoma Based on Smart Healthcare. J Healthc Eng (2022) 2022:5914541. doi: 10.1155/2022/5914541 35028121PMC8752226

[29] WuHLiuBChenZLiGZhangZ. MSC-Induced lncRNA HCP5 Drove Fatty Acid Oxidation Through miR-3619-5p/AMPK/PGC1alpha/CEBPB Axis to Promote Stemness and Chemo-Resistance of Gastric Cancer. Cell Death Dis (2020) 11(4):233. doi: 10.1038/s41419-020-2426-z 32300102PMC7162922

[30] TangXLiuBZhangCTangWLiangSXiaoY. SENP2 Reduces Hepatocellular Carcinoma Stemness and Improves Sorafenib Sensitivity Through Inactivating the AKT/GSK3beta/CTNNB1 Pathway. Front Oncol (2021) 11:773045. doi: 10.3389/fonc.2021.773045 34950583PMC8688154

[31] da CostaVRAraldiRPVigerelliHD'AmelioFMendesTBGonzagaV. Exosomes in the Tumor Microenvironment: From Biology to Clinical Applications. Cells (2021) 10:(10). doi: 10.3390/cells10102617 PMC853389534685596

[32] LiCTeixeiraAFZhuHJTen DijkeP. Cancer Associated-Fibroblast-Derived Exosomes in Cancer Progression. Mol Cancer (2021) 20(1):154. doi: 10.1186/s12943-021-01463-y 34852849PMC8638446

[33] BaLXueCLiXZhangMYangYHanQ. Gastric Cancer Cell-Derived Exosomes Can Regulate the Biological Functions of Mesenchymal Stem Cells by Inducing the Expression of Circular RNA Circ_0004303. Stem Cells Dev (2021) 30(16):830–42. doi: 10.1089/scd.2021.0059 34098776

[34] BiswasSMandalGRoy ChowdhurySPurohitSPayneKKAnadonC. Exosomes Produced by Mesenchymal Stem Cells Drive Differentiation of Myeloid Cells Into Immunosuppressive M2-Polarized Macrophages in Breast Cancer. J Immunol (2019) 203(12):3447–60. doi: 10.4049/jimmunol.1900692 PMC699491931704881

[35] WangSSuXXuMXiaoXLiXLiH. Exosomes Secreted by Mesenchymal Stromal/Stem Cell-Derived Adipocytes Promote Breast Cancer Cell Growth *via* Activation of Hippo Signaling Pathway. Stem Cell Res Ther (2019) 10(1):117. doi: 10.1186/s13287-019-1220-2 30971292PMC6458638

[36] YangYPNguyenPNNMaHIHoWJChenYWChienY. Tumor Mesenchymal Stromal Cells Regulate Cell Migration of Atypical Teratoid Rhabdoid Tumor Through Exosome-Mediated Mir155/SMARCA4 Pathway. Cancers (Basel) (2019) 11:(5). doi: 10.3390/cancers11050720 PMC656312631137686

[37] GuHYanCWanHWuLLiuJZhuZ. Mesenchymal Stem Cell-Derived Exosomes Block Malignant Behaviors of Hepatocellular Carcinoma Stem Cells Through a lncRNA C5orf66-AS1/microRNA-127-3p/DUSP1/ERK Axis. Hum Cell (2021) 34(6):1812–29. doi: 10.1007/s13577-021-00599-9 34431063

[38] LiYHLvMFLuMSBiJP. Bone Marrow Mesenchymal Stem Cell-Derived Exosomal MiR-338-3p Represses Progression of Hepatocellular Carcinoma by Targeting ETS1. J Biol Regul Homeost Agents (2021) 35(2):617–27. doi: 10.23812/20-638-A 33884828

[39] PezoulasVCHazapisOLagopatiNExarchosTPGoulesAVTzioufasAG. Machine Learning Approaches on High Throughput NGS Data to Unveil Mechanisms of Function in Biology and Disease. Cancer Genomics Proteomics (2021) 18(5):605–26. doi: 10.21873/cgp.20284 PMC844176234479914

[40] SunEJWankellMPalamuthusingamPMcFarlaneCHebbardL. Targeting the PI3K/Akt/mTOR Pathway in Hepatocellular Carcinoma. Biomedicines (2021) 9:(11). doi: 10.3390/biomedicines9111639 PMC861561434829868

[41] Deldar Abad PaskehMMirzaeiSAshrafizadehMZarrabiASethiG. Wnt/beta-Catenin Signaling as a Driver of Hepatocellular Carcinoma Progression: An Emphasis on Molecular Pathways. J Hepatocell Carcinoma (2021) 8:1415–44. doi: 10.2147/JHC.S336858 PMC863046934858888

[42] Gonzalez-SanchezEVaqueroJFernandez-BarrenaMGLasarteJJAvilaMASarobeP. The TGF-Beta Pathway: A Pharmacological Target in Hepatocellular Carcinoma? Cancers (Basel) (2021) 13:(13). doi: 10.3390/cancers13133248 PMC826832034209646

[43] AnYJiangJZhouLShiJJinPLiL. Peroxiredoxin 1 Is Essential for Natamycin-Triggered Apoptosis and Protective Autophagy in Hepatocellular Carcinoma. Cancer Lett (2021) 521:210–23. doi: 10.1016/j.canlet.2021.08.023 34428517

[44] WangNFengYTanHYCheungFHongMLaoL. Inhibition of Eukaryotic Elongation Factor-2 Confers to Tumor Suppression by a Herbal Formulation Huanglian-Jiedu Decoction in Human Hepatocellular Carcinoma. J Ethnopharmacol (2015) 164:309–18. doi: 10.1016/j.jep.2015.02.025 25700642

[45] LebeaupinCBlancMValleeDKellerHBailly-MaitreB. BAX Inhibitor-1: Between Stress and Survival. FEBS J (2020) 287(9):1722–36. doi: 10.1111/febs.15179 PMC720297631841271

[46] LiaoYQiuZBaiL. Mir302d3p Regulates the Viability, Migration and Apoptosis of Breast Cancer Cells Through Regulating the TMBIM6mediated ERK Signaling Pathway. Mol Med Rep (2021) 24:(6). doi: 10.3892/mmr.2021.12493 PMC854893934651659

[47] LuBLiYLiHZhangYXuJRenL. Bax Inhibitor-1 Is Overexpressed in Non-Small Cell Lung Cancer and Promotes Its Progression and Metastasis. Int J Clin Exp Pathol (2015) 8(2):1411–8.PMC439628825973025

[48] WangXTianLLiYWangJYanBYangL. RBM15 Facilitates Laryngeal Squamous Cell Carcinoma Progression by Regulating TMBIM6 Stability Through IGF2BP3 Dependent. J Exp Clin Cancer Res (2021) 40(1):80. doi: 10.1186/s13046-021-01871-4 33637103PMC7912894

[49] JinZPiaoLHSunGCLvCXJingYJinRH. Long Non-Coding RNA Plasmacytoma Variant Translocation 1 (PVT1) Promotes Glioblastoma Multiforme Progression *via* Regulating miR-1301-3p/TMBIM6 Axis. Eur Rev Med Pharmacol Sci (2020) 24(22):11658–65. doi: 10.26355/eurrev_202011_23810 33275233

[50] WilsonMMWeinbergRALeesJAGuenVJ. Emerging Mechanisms by Which EMT Programs Control Stemness. Trends Cancer (2020) 6(9):775–80. doi: 10.1016/j.trecan.2020.03.011 32312682

[51] XueCLiGLuJLiL. Crosstalk Between circRNAs and the PI3K/AKT Signaling Pathway in Cancer Progression. Signal Transduct Target Ther (2021) 6(1):400. doi: 10.1038/s41392-021-00788-w 34815385PMC8611092

[52] LiuGOuyangXSunYXiaoYYouBGaoY. The miR-92a-2-5p in Exosomes From Macrophages Increases Liver Cancer Cells Invasion *via* Altering the AR/PHLPP/p-AKT/beta-Catenin Signaling. Cell Death Differ (2020) 27(12):3258–72. doi: 10.1038/s41418-020-0575-3 PMC785314932587378

